# A Meta-Analysis of the Influence of Tumor Necrosis Factor-*α*-308 Gene Polymorphism on Liver Cirrhosis

**DOI:** 10.1155/2022/9764770

**Published:** 2022-03-19

**Authors:** Chang Liu, Songtao Yang

**Affiliations:** Department of Gastroenterology, The First People's Hospital of Chong Qing Liang Jiang New Area, Chongqing 401121, China

## Abstract

Cirrhosis is an active hepatic inflammation process of the liver considered as the serious phase of different liver injuries. Epidemiological studies have evaluated the possible association between TNF-*α*-308G/A gene polymorphism and liver cirrhosis. In this study, we have furthered the study to assess the exact association of TNF-*α*-308G/A gene polymorphism with liver cirrhosis susceptibility by integrating all available data. Eligible case-control studies were carried out from the establishment of the project to September 2021. Published literature from multiple databases was retrieved, collected, and analyzed by two investigators independently. Odds ratios (ORs) and 95% confidence intervals (CIs) were calculated for every study. Review Manager 5.2 and Stata 15.0 software were used for meta-analysis and stability was assessed by both subgroup analysis and sensitivity analysis. Begg's funnel plot and Egger's regression across the studies were also explored. We examined 22 case-control studies with 2683 cirrhosis patients and 2905 normal controls in four genetic models (GA vs. GG: OR = 0.95, 95%CI: (0.70, 1.30); AA vs. GG: OR = 1.11, 95% CI: (0.66, 1.85), GA + AA vs. GG: OR = 1.00, 95% CI: (0.73, 1.37); AA vs. GA + GG: OR = 1.07, 95%CI: (0.70,1.63)). TNF-*α*-308G/A gene polymorphism was relatively independent, and the results did not show a significant difference between the two groups. In the subgroup analysis by etiological classification of liver cirrhosis, cirrhosis after HCV infection was positively associated with the risk of TNF-*α*-308G/A polymorphism (AA vs. GG: OR = 3.02, 95% CI: (1.15, 7.88), AA vs. GA + GG: OR = 2.68, 95% CI: (1.04, 6.95)). The meta-analysis showed TNF-*α*-308G/A gene polymorphism might not have affected susceptibility for liver cirrhosis. Nevertheless, further and well-designed studies were needed to confirm the findings.

## 1. Introduction

Cirrhosis is an active hepatic inflammation process of the liver that is considered as the serious phase of different liver injuries [1]. It is characterized by diffuse fibrosis, pseudolobule formation, and proliferation of blood vessels inside and outside the liver. Morbidity and mortality resulting from cirrhosis in more developed countries were increasing, making it rank the 14th most common cause of death worldwide and fourth in Europe [2]. The main causes of cirrhosis in the world were alcohol seminal liver disease, nonalcoholic fatty liver disease, and chronic viral infections. Other causes include primary biliary cirrhosis (PBC), autoimmune hepatitis, primary sclerosing cholangitis, and genetic and metabolic diseases, such as Wilson's disease and hemochromatosis. A complex gene regulatory network underlying immune response processes might play an important role in the development and progression of liver cirrhosis [3].

Risk factors, such as age, gender, alcohol, and obesity, failed to explain all the clinically evident differences and also varied in patients. The advent of new genomic technologies and the decreasing cost of genotyping, together with multiple studies, enabled us to put much emphasis on the importance of genetic predisposition in different liver diseases. We realized that single nucleotide polymorphisms (SNPs) could not be neglected in determining fibrosis risk [4].

TNF-*α* is a kind of cytokine with important immunoregulatory function and is involved in the inflammatory response. The TNF-*α* gene lies in the class III region of the major histocompatibility complex (MHC). According to the gene location inference, the location of the gene polymorphism might be related to immune infections [5]. The common allele at locus –308 had been indicated as TNF-*α*-308G, or TNF1, and the uncommon allele as TNF-*α*-308A, or TNF2. The TNF2 promoter fragment functions were used as a powerful transcriptional activator [6].

A series of studies have been conducted to research the possible relationship between TNF gene statistical analysis polymorphisms and liver cirrhosis. Several TNF alleles and haplotypes which were defined by TNF−308G/A dimorphic sequences were observed [5]. Polymorphisms in the TNF-*α* promoter appeared to be associated with variability in the histological severity of chronic hepatitis C infection [7]. TNF-*α* reduced AMP-activated protein kinase (AMPK) activity, which could contribute to the development of NAFLD [8]. Increased TNF-*α* production induced by HBV and HCV leads to hypoalbuminemia [9]. Gordon showed a low prevalence of the TNF allele in patients with PBC. A distinct genetic risk of developing PBC in the Italian population was found with no interaction between the HLA and TNF alleles [10]. TNF- *α* is the first cytokine produced by the inflammatory response mechanism, which jointly promotes the proliferation and fiber proliferation of hepatic stellate cells, inhibits the growth of hepatocytes, prevents the regeneration of hepatocytes, and participates in the formation and development of cirrhosis [11]. The result was obtained by meta-analysis to evaluate the relationship between the TNF-*α*-308G/A polymorphisms and the risk of liver cirrhosis.

## 2. Methods

This systematic review and meta-analysis were conducted following the Preferred Reporting Items for Systematic Reviews Results and Meta-analysis (PRISMA) guidelines.

### 2.1. Data Sources

Comprehensive systematic electronic search studies were published from building databases to September 2021. Published literature from PubMed, Embase, Web of Science, Google Scholar, Chinese National Knowledge Infrastructure (CNKI), and Wanfang Data were retrieved, collected, and analyzed by two investigators independently. The search keywords were as follows: (“liver cirrhosis” or “cirrhosis” or “hepatic cirrhosis” or “primary biliary cirrhosis (PBC),” “hepatitis C virus (HCV) liver cirrhosis,” “alcoholic liver cirrhosis (ALC),” “hepatitis B virus (HBV) liver cirrhosis,” “hereditary hemochromatosis”) and (“TNF-*α*-308G/A” or “gene polymorphism” or “TNF” or “tumor necrosis factor” or “polymorphism” or “variant”). Moreover, we also collected literature through references lists of the relevant.

### 2.2. Inclusion Criteria

The inclusion criteria of this meta-analysis were as follows: (1) a case-control study or nested case-control study expressed in published journals; (2) comparing the risk of TNF-*α*-308G/A in susceptibility with liver cirrhosis; (3) the data from the article about genotype frequency of cases and controls were calculated; and (4) in the case-control group, there were the total number and genotype distribution and frequency with the Hardy–Weinberg balance (*P* < 0.05 that did not conform to the Hardy–Weinberg balance).

### 2.3. Exclusion Criteria

The exclusion criteria were as follows: (1) reviews and meta-analyses; (2) duplicate studies; (3) irrelevant literature; (4) studies without controls, or studies that did not show genotype frequency were also excluded from this meta-analysis; (5) liver cirrhosis was accompanied by serious complications or liver cancer; and (6) the control group was not healthy people.

### 2.4. Data Extraction

Two authors extracted the following data independently using the inclusion and exclusion criteria set by our group. The following information was collected from each study: the first name of the author, published time, country in which the study was launched, ethnicity, the number of cases and controls, allele frequency, types of study design, sample size, and types of cirrhosis. In case-control, the genotype frequency was consistent with the Hardy-Weinberg balance. We advocated solving the dispute by discussion, instead of our own decisions.

### 2.5. Inclusion of Research Bias Risk Assessment

The New Castle Ottawa scale was used to evaluate the risk of bias. Through the selection of research objects, comparability between groups, and exposure factors, 8 items were included in the study, with a full score of 9 points, 0–4 points for low-quality studies, and 5–9 points for high-quality studies.

### 2.6. Statistical Analysis

The odds ratio (OR) with 95% CI statistical methods could be used as the important method to calculate the association between the TNF-*α*-308 polymorphisms and liver cirrhosis for each study. In view of the heterogeneity of the results, heterogeneity was assessed by the I^2^ statistic, where in I^2^<50% indicates minor heterogeneity, for which a fixed effect model was used, and I^2^ > 50 indicates large heterogeneity, for which a random effect model was used. The results of heterogeneity were affected by many factors, such as different types of cirrhosis, a limited number of patients, and so on. Subgroup analysis was performed according to the racial population and different types of cirrhosis. The funnel plot, Begg's funnel plot, and Egger's regression tests were used to analyzing publication bias. Analyses were performed by the software Review Manager 5.2 and STATA 15.0 *P*values. *P* < 0.5 was considered statistically significant.

## 3. Results

A comprehensive search of retrieved websites generated a total of 542 references based on the search strategy, including 65 relevant Chinese articles and 477 relevant English articles. 453 studies were excluded according to the first screening of titles, abstract diagrams, and full-text reading. 89 studies were retrieved for more details and excluded the overview, meta-analysis, and basic research. At this stage, 28 research literature studies were reviewed again. Based on the preset inclusion and exclusion criteria, 6 articles were excluded for lack of original data or case-control data. Finally, a total of 22 studies with 2683 cirrhosis patients and 2905 normal controls were included in the quantitative analysis [10, 12–31] (Figure 1). 7 Chinese articles and 15 English articles were included in the final. Meanwhile, the types of cirrhosis were 10 articles of PBC, 6 articles of hepatitis B cirrhosis, 3 articles of hepatitis C cirrhosis, 2 articles of alcoholic cirrhosis, and 1 article of homochromatic cirrhosis. There were 7 races from Asians, 10 Europeans, 2 Americans and 3 Africans. The characteristics of selected studies are summarized in Table 1.

### 3.1. Data Analysis

TNF-*α*-308G/A polymorphism and the risk of liver cirrhosis are presented in Table 2. On the whole, the results showed that the TNF-308G/A polymorphism was relatively independent of liver cirrhosis, which was not associated with the risk of liver cirrhosis under a random-effects model. Heterogeneity for all studies was explored, and the test value of *χ*^2^ was about *P* ≤ 0.1 in a random-effect model. There was statistical heterogeneity in four genetic models (dominant, recessive, codominant, and overdominance). For GA vs. GG (*P* < 0.00001; I^2^ = 73%): OR = 0.95, 95% CI = 0.70–1.30, and test for overall effect: *Z* = 0.31(*P* = 0.76). For AA vs. GG (*P* < 0.0005; I^2^ = 59%): OR = 1.11, 95% CI = 0.66–1.85, and test for overall effect: *Z* = 0.38 (*P* = 0.70). For GA + AA vs. GG (*P* < 0.00001; I^2^ = 78%): OR = 1.00, 95% CI = 0.73–1.37, and test for overall effect: *Z* = 0.00 (*P* = 1.00). For AA vs. GA + GG (*P* < 0.002; I^2^ = 54%): OR = 1.07, 95% CI = 0.70–1.63, and test for overall effect: *Z* = 0.29 (*P* = 0.77).

In the further subgroup analysis based on ethnology, TNF-*α*-308G/A gene polymorphism was relatively independent of liver cirrhosis risk including Asians, Africans, Americans, and Europeans in all genetic models. However, the results of subgroup analysis by etiological classification of liver cirrhosis were different. Cirrhosis after HCV infection was positively associated with the risk of TNF-*α*-308G/A polymorphism. For AA vs. GG (*P* = 0.518; I^2^ = 0.0%): OR = 3.02, 95% CI = 1.15–7.88. For AA vs. GA + GG (*P* < 0.00001; I^2^ = 0.645%): OR = 2.68, 95% CI = 1.04–6.95. Other subgroup analyses by classification of liver cirrhosis did not reveal a significant association with TNF -308G/A gene polymorphism (ALC, PBC, HHC, HHC, and HBV). The partial forest plots are shown in Figures 2 and 3.

### 3.2. Sensitivity Analysis

Sensitivity analysis was carried out by repeating the meta-analysis sequentially and excluding one study at a time to evaluate the degree to which each individual study affected the overall OR. Our previous sensitivity analysis about the TNF-*α*-308G/A polymorphism and liver cirrhosis risk under all models in both the overall analysis and subgroup analysis showed the results did not alter substantially under any genetic models. Since the estimated pooled ORs were not affected by the data, this aspect suggested that our results were stable. TNF-*α*-308G/A gene polymorphism (GA vs. GG) sensitivity analysis is shown in Figure 4.

### 3.3. Bias Diagnostics

We observed that the funnel of Begg's funnel plots were basically symmetrical. Using Egger's regression, no publication bias could be detected for studies published on TNF-*α*-308G/A gene polymorphism (GA vs. GG, *P* = 0.39; AA vs. GG, *P* = 0.98; GA + AA vs. GG, *P* = 0.11; and AA vs. GA + GG, *P* = 1.33). *P* < 0.05 suggested the presence of publication bias. As expected, no significant publication bias was detected by Begg's funnel plot for the association between TNF- *α*-308G/A gene polymorphism and liver cirrhosis expected (GA vs. GG, *P* = 0.675; AA vs. GG, *P* = 0.261; GA + AA vs. GG, *P* = 0.866; and AA vs. GA + GG, *P* = 0.199) (Figure 5).

## 4. Discussion

Cirrhosis is an active hepatic inflammation process of the liver. It is characterized by diffuse fibrosis, pseudolobule formation, and proliferation of blood vessels inside and outside the liver. TNF- *α* is closely related to the occurrence, development, and outcome of liver diseases. TNF- *α* is the first cytokine produced by the inflammatory response mechanism, which jointly promotes the proliferation and fiber proliferation of hepatic stellate cells, inhibits the growth of hepatocytes, prevents the regeneration of hepatocytes, and participates in the formation and development of cirrhosis [11]. Located in the center of the major histocompatibility complex part TNF- *α*, there are probably huge quantities of other immune genes around [32]. TNF- *α* gene regulation has a considerable challenge, as it can be used as innate immunity and inflammatory pathology agent. In recent years, there has been an increasing number of studies on the relationship between TNF- *α* and cirrhosis, such as PBC, hepatitis B, alcoholic hepatitis, and hepatitis C. The research literature between on liver cirrhosis caused by HBV, PBC, and TNF- *α*-308 gene were various. In our included literature, TNF- *α* promoter polymorphism (G-308A and G-238A) and alleles of HLA class II (HLA-DRB1) might be associated with the occurrence and severity of PBC in Italians. We realized that single nucleotide polymorphisms (SNPs) could not be neglected in determining fibrosis risk. TNF- *α* is the host defense key mediator of various kinds of viruses and inflammatory response. Opinions of meta-analysis report were inconsistent. One meta-analysis published in 2011 on the association between TNF- *α* -308 polymorphism and cirrhosis risk failed to present as many cases as possible. The results were consistent with our study [33]. Other studies, such as the one from Bao Dong Qin who published a meta-analysis about the association of TNF- *α* polymorphisms with PBC risk also presented no significant associations [34]. The literature about TNF- *α*-308 gene polymorphisms and hepatitis C virus infection meta-analysis might have no effect on susceptibility to HCV infection and virus clearance [35]. Our meta-analysis was to identify the relationship between TNF-*α* -308G/A polymorphism and liver cirrhosis risk. Finally, this meta-analysis covered 22 case-control studies, 2683 cirrhosis patients, and 2905 normal controls. HBV-related studies were mostly found in the Chinese population, and PBC-related studies were limited to the Caucasian population, without a unified review of the population. Based on our notion, our study was more about investigation of the worldwide evidence about TNF-*α*-308 polymorphism and cirrhosis risk.

Based on previous studies, this study expanded the sample size, and the meta-analysis method was used in the comprehensive evaluation and analysis of TNF- *α* -308 gene polymorphism on liver cirrhosis. No significant correlation was found between TNF-*α* -308G/A polymorphism and liver cirrhosis risk in all comparisons of GA vs. GG; GA + AA vs. GG; AA vs. GA + GG; AA vs. GG. Cirrhosis after HCV infection was positively associated with the risk of TNF-*α*-308G/A polymorphism. However, the results were related to genetic polymorphism and the small sample size of the HCV subgroup, so it did not change the overall result. A single study method was deleted each time to reﬂect the influence of the individual data-set to the pooled ORs. All this proves the fact that the results would not be altered by the change of individual studies.

The part of the presence of heterogeneity in all genetic models might be obtained through sensitivity analysis and subgroup, eliminating any document for the reason of the heterogeneity. Finally, the significance of these results was the same and did not vary with the abovementioned statement. We analyzed the causes of heterogeneity and found that it mainly lay in different countries, races, gene types, and the etiology of liver cirrhosis. In this paper, we used Egger's test for the qualitative and quantitative assessment of publication bias tips. Heterogeneity did not affect the results of publication bias, which increased the statistical power.

## 5. Conclusion

There were some limitations to the research which are as follows: (1) only the published Chinese and English literature was included, which might lead to selection bias; (2) all the literature were case-control studies, which were highly heterogeneous and lacked the support of higher quality clinical trial research; (3) the original literature only involved European, Asian, African, and American populations, but not the Oceania population, and there were only fewer data in Africa and America population; and (4) more PBC and HCV studies, less HCV/HHC/ALC population. In spite of the above limitations, all 22 articles conformed to HWE's law of equilibrium. The result of the meta-analysis was reliable, which means there was no significant publication bias indicated by Begg's funnel diagram. Nevertheless, larger and well-designed studies were needed to confirm the findings. Our future research is to further study these limitations.

## Figures and Tables

**Figure 1:** The flowchart of research selection.

**Figure 2:** Forest plot of studies using a random effects model (dominant model GA vs. GG).

**Figure 3:** Subgroup analysis by forest plot of cirrhosis type using a random effects model (dominant model AA + GA vs. GG).

**Figure 4:** TNF- *α*-308G/A gene polymorphism (GA vs. GG) sensitivity analysis.

**Figure 5:** Begg's funnel plot for publication bias in the studies (GA vs. GG).

**Table 1:** Main characteristics of studies for meta-analysis.

Study	Area	Ethnology	Cirrhosis type	Sample size (case and control)	Genotype case (GG/GA/AA)	Distribution case (GG/GA/AA)	NOS score (sub)
Tanaka A	Italian	European	PBC	71/133	56/14/1	109/24/0	8
Bahr MJ	German	European	HCV	50/200	38/9/3	139/55/6	8
Bathgate AJ	Scotland	European	PBC	61/8	34/23/4	0/4/4	8
Bernal W	England	European	PBC	109/126	46/44/20	89/35/2	8
Bittencourt	Brazilian	American	PBC	57/83	48/9/0	63/19/1	7
Jones DEJ	England	European	PBC	168/145	111/53/4	87/49/9	7
Juran BD	Canadian	American	PBC	360/404	236/114/10	289/105/10	6
Juran BD	Canadian	American	PBC	506/357	24/121/361	12/76/269	6
Gordon	England	European	PBC	91/209	66/20/5	122/78/9	8
Nguyen-Khac	French	European	ALC	45/47	26/13/6	21/25/1	7
NiroGA	Italian	European	PBC	107/141	90/16/1	115/25/1	7
Osterreicher CH	Austrian	European	HHC	55/94	44/10/1	74/19/1	6
Pastor	Spanish	European	ALC	65/90	45/19/1	69/19/2	8
Radwan	Egyptian	African	HCV	152/160	108/40/4	136/24/0	8
SGHAIER Ikram	Tunisians	African	HBV	200/36	80/72/48	11/14/11	8
Talaat	Egyptian	African	HCV	45/45	25/13/7	39/3/3	8
Fan	Chinese	Asian	PBC	58/160	52/6/0	133/27/0	7
Jiang	Chinese	Asian	HBV	169/119	145/18/6	71/38/10	7
LiH	Chinese	Asian	HBV	30/40	23/7/0	38/2/0	6
Cheng YQ	Chinese	Asian	HBV	106/108	85/21/0	97/11/0	6
Wu YD	Chinese	Asian	HBV	150/150	96/15/39	84/22/44	7
Zhang P	Chinese	Asian	HBV	28/50	25/2/1	47/2/1	7

**Table 2:** Summary of pooled ORs and 95%CI for TNF-*α*-308G/A gene polymorphism and subgroup analyses.

	(GA vs. GG)		(AA vs. GG)		(GA + AA vs. GG)		(AA vs. GA + GG)	
	OR, 95% CI P, I^2^		OR, 95% CI P, I^2^		OR, 95% CI P, I^2^		OR, 95% CI P, I^2^	
Total	0.95 (0.70,1.30)	*P* < 0.00001; I^2^ = 73%	1.11 (0.66,1.85)	*P* < 0.0005; I^2^ = 59%	1.00 (0.73,1.37)	*P* < 0.00001; I^2^ = 78%	1.07 (0.70,1.63)	*P* = 0.002; I^2^ = 54%
European	0.86 (0.58,1.27)	*P* = 0.002; I^2^ = 65%	1.19 (0.42,3.37)	*P* = 0.001; I^2^ = 67%	0.93 (0.60,1.43)	*P* < 0.00001; I^2^ = 74%	0.43 (0.41,4.99)	*P* = 0.0002; I^2^ = 73%
American	0.95 (0.57,1.59)	*P* = 0.11; I^2^ = 54%	0.70 (0.28,1.77)	*P* = 0.25; I^2^ = 29%	0.91 (0.53,1.57)	*P* = 0.09; I^2^ = 59%	0.84 (0.63, 1.12)	*P* = 0.75; I^2^ = 0%
African	2.97 (0.56,15.64)	*P* = 0.002; I^2^ = 83%	2.08 (0.39,11.23)	*P* = 0.03; I^2^ = 71%	1.92 (0.67, 5.53)	*P* = 0.003; I^2^ = 82%	1.68 (0.44, 6.36)	*P* = 0.09; I^2^ = 58%
Asian	0.95 (0.38,2.35)	*P* = 0.0001; I^2^ = 82%	0.60 (0.28,1.30)	*P* = 0.2; I^2^ = 37%	0.97 (0.43,2.19)	*P* = 0.0001; I^2^ = 83%	0.75 (0.48, 1.18)	*P* = 0.37; I^2^ = 0%
PBC	0.90 (0.63,1.28)	*P* = 0.002; I^2^ = 65%	0.80 (0.22,2.88)	*P* = 0.0001; I^2^ = 82%	0.90 (0.59, 1.35)	*P* = 0.0001; I^2^ = 76%	0.98 (0.45, 2.10)	*P* = 0.0008; I^2^ = 70%
HCV	1.85 (0.58,5.88)	*P* = 0.04; I^2^ = 82%	3.02 (1.15,7.88)	*P* = 0.5; I^2^ = 0%	1.96 (0.71, 5.40)	*P* = 0.004; I^2^ = 82%	2.68 (1.04, 6.95)	*P* = 0.63; I^2^ = 0%
ALC	0.82 (0.23,2.92)	*P* = 0.03; I^2^ = 79%	2.08 (0.34,12.73)	*P* = 0.27; I^2^ = 19%	0.95 (0.39, 2.31)	*P* = 0.10; I^2^ = 62%	2.36 (0.24, 23.38)	*P* = 0.16; I^2^ = 50%
HBV	0.78 (0.32,1.92)	*P* = 0.002; I^2^ = 76%	0.64 (0.41,0.99)	*P* = 0.36; I^2^ = 7%	0.98 (0.45, 2.15)	*P* = 0.0001; I^2^ = 83%	0.74 (0.50, 1.10)	*P* = 0.57; I^2^ = 0%

## Data Availability

All the data generated or analyzed during this study are included in this article. Further enquiries can be directed to the corresponding author.
